# Bionic Anti-Slipping Crimping Structure for Industrial Hose Assembly Inspired by Ruminant Molars

**DOI:** 10.1155/2022/5632586

**Published:** 2022-03-29

**Authors:** Xianghua Zheng, Cong Cheng, Wei Yuan

**Affiliations:** ^1^School of Intelligent Manufacturing, Chengdu Technological University, Chengdu 611730, China; ^2^Northwest Industries Group Co., Ltd., Xi'an 710043, China; ^3^Sichuan Institute of Geological Engineering Investigation Group Co., Ltd., Chengdu 610032, China

## Abstract

It is highly desirable to improve the anti-slipping stability of the crimping structure for a reliable connection. This study innovatively presents a biomimetic strategy for designing a high-performance crimping structure for industrial hose assembly based on evidence that the special infundibulum dentis structure on the occlusal surface of ruminant molars has the potential of anti-slippage and can also reduce the risk of stress concentration. Utilizing reverse engineering technology, the three-dimensional (3D) digital model of the bovine molar was built as a representative prototype, and then corresponding characteristics of the infundibulum dentis were extracted with a fitting method for the bionic design of the crimping structure. Numerical simulations and experimental results both indicate that the bionic crimping structure has high resistance to slippage of hose body compared with the traditional type, and further, the formation mechanism of bionic anti-slipping performance was discussed.

## 1. Introduction

The hose assembly is formed by crimping a hose body and a connecting joint for transporting fluid with a certain pressure and flow rate. It is an important pipeline component in the fluid transmission and control system, widely used in processing equipment, construction machinery, transportation machinery, mining machinery, etc. [1–3]. However, in actual use, it is often exposed that the hose assembly bursts and leaks at the crimping end, and even the hose slips off from the crimp due to the unreasonable crimping structure, causing serious security threats [4–6]. As shown in Figure 1, the crimping structure referring to the shape and size of the inner teeth of the sleeve and the outer teeth of the core rod directly determines the crimping strength and sealing performance of the hose after crimping. The traditional design of the crimping structure often depends on engineering experience; the tribological design theory is lagging, and the collaborative design mechanism is not clear, resulting in poor crimping performance as mentioned above. Therefore, it is necessary to improve the crimping structure and performance for increasing the reliability of the hose assembly.

Learning from nature seems to be a perfect solution. Natural selection, as everyone knows, created various near-perfect geometries and functional mechanisms in teeth evolution, to adapt to different conditions of service. In general, they function efficiently in terms of penetrating or cutting the feed with less energy based on corresponding morphological characteristics as cusps and crests, respectively [7, 8]. Natural teeth have become an important biospecimen, and the research progress in bionics of teeth structure has been reported successively, with the development of bionic tribology. Recently, a biomimetic blade for corn harvester designed by Tian et al. (2017) based on the cutting tooth profile curve of the *B. horsfieldi* palate was found to have strong cutting ability and good cutting quality, and it was proved that the average maximum cutting force and cutting energy consumption can be reduced obviously [9]. Zhang et al. developed a bionic imprinting toothed wheel inspired by the foreleg end-tooth of soil-burrowing dung beetle, eventually reducing the forward resistance and expanding the volume of imprinted microbasin [10]. To improve the crushing performance in powder processing, bionic grinding heads based on natural friction pairs of bovine teeth were presented by Wang et al., enabling a higher reduction ratio and lower working temperature effectively [11, 12]. The above typical bionic structures have achieved good application effects in either cutting or grinding tools, whereas transferring geometric characteristics of natural teeth to crimping structures is rare.

It is noteworthy that the infundibulum dentis, a funnel-shaped depression structure on the surface of ruminant molars (see Figure 2), is of particular importance in holding feed: ruminants feed more on crude fiber and need more chewing activities; then the presence of infundibulum dentis by convergent evolution enhances the anti-sliding stability of the tooth structure; thus, the feed can be fully ground between its powerful molars when trapped in it [13–16]. Vollmerhaus et al. once studied the various geometries of the infundibulum dentis during the life cycle of horses and inferred that this construction results in a good grip of the occlusal surface and the efficiency of ingestion [17]. Wang et al. further showed its holding function in the chewing simulation of bovine molars and developed biomimetic high-performance grinding heads, which has been demonstrated experimentally [11, 12]. Also, Weimer et al. indicated the potential for biomimetic application of ruminant infundibulum dentis to holding design in a bioreactor [18]. Those all provide clues for the bionic anti-slipping design of the crimping structure. On the other hand, the most stable occlusal mode for both human and animal teeth is known as the intercuspid position (ICP), as illustrated in Figure 3 [19]. This occlusal contact occurs between the cusp and the fossa and is another manifestation of convergent evolution. It contributes to transmitting the occlusal load during clenching in all directions perpendicular to the inclined plane of the tooth cusp, thereby avoiding the concentration of local occlusal force caused by two-point contact, as well as damage to the tooth and periodontal tissue during occlusion [19–21]. From here we can see that the vertical occlusion of teeth is highly similar to the crimping process of industrial hose; hence, developing a bionic crimping structure inspired by the surface topography and functional principle of typical teeth may be an effective way to achieve high-reliability crimping.

Bovine is a typical representative of ruminants, and the infundibulum dentis on their molars shows a high degree of structural and functional similarity to the crimping structure. Moreover, the properties of the materials processed by occluding and crimping are similar to a certain extent. Accordingly, this article focuses on the prototype of bovine molars, and the geometric characteristics and functional principles existing in this natural friction pair were abstracted and imitated from the perspective of convergent evolution. Then, a bioinspired crimping structure with good anti-slipping performance was developed for industrial hose assembly and demonstrated by numerical simulations and experiments compared to the traditional one.

## 2. Materials and Methods

### 2.1. Sample Collection, Handling, and Modeling

The bovine mandibular first molar as the selected component was separated from adult cattle in a local abattoir and then sterilized with 75% alcohol, washed with distilled water, and sprayed with a white developer on its surface. For morphology measurement, the point cloud data of the bovine molar was acquired using the 3D laser scanner, and then the CAD model of bovine molar was reconstructed assisted with Geomagic Studio, a reverse engineering software, after data reduction, noise reduction, and other preprocessing, as well as package processing, polygon editing, and NURBS surface construction, sequentially for the point cloud as shown in Figure 4 [22–24]. It provides a digital foundation for the geometric extraction of the bionic coupling element.

### 2.2. Extraction of Biological Coupling Elements

In this section, the infundibulum dentis was selected as the biological coupling element for designing bioinspired crimping structures based on the functional and structural similarities, and then its feature was extracted by fitting method with CAD software.  Figure 2 presents the extracted sectional contour of the infundibulum dentis. In the coronal plane through the infundibulum cusp, the infundibulum dentis was characterized by using straights to match the profile of the infundibulum groove, forming an included angle *α* and a positive rake angle *β* to describe the biological coupling element.

### 2.3. Design and Performance Simulation of Bioinspired Crimping Structure

According to ICP, the most stable occlusal mode for natural teeth, we proposed a cusp-to-fossa crimping form and developed a crimping surface structure coupled with the characteristics of the infundibulum dentis of the bovine molar extracted in Section 2.2.

To examine its crimping performance, comparative finite element analyses were conducted with the traditional cusp-to-cusp structure. In the simulation, the hose body was assumed as an anisotropic and elastic hollow cylinder with rubber properties, and its elastic modulus and Poisson's ratio were set to 6.11N/m^2^ and 0.49, respectively. Due to the circular symmetry of the crimping structure in action, the inner teeth of the sleeve and the outer teeth of the core rod were considered as a pair of rigid toothed racks with Q235 steel properties. The corresponding elastic modulus and Poisson's ratio were 210GPa and 0.27, respectively. Furthermore, simulations only focus on a shaft section through X-Y to simplify the analysis seen in Figure 5, and the coefficient of friction between them is set to 0.7. The geometrically nonlinear simulation process of the crimping structure is as follows: the hose body was fixed, and 2-mm displacement constraint along the ±X direction was first introduced to the inner/outer teeth, respectively, to simulate the crimping process; then 2-mm displacement constraint in the -Y direction was simultaneously applied to them to simulate the working process. For the statistics of the analysis results, the Mises stress and maximum principal strain were both selected as indicators of the crimping performance (see Figures 6 and 7).

### 2.4. Crimping Performance Test

To evaluate the anti-slip performance of the crimping structure, the control variable method was applied in the comparative tensile tests for crimped materials based on the electronic universal testing machine.  Figure 8 shows the tensile test platform. The aluminum bionic and traditional crimping parts seen in Figure 9 were first manufactured with CNC milling technology. The crimped material, the rubber band was made with the size of 3(THK) × 30(W) × 400(L) mm, and one end was attached by clamps and can move with the transverse beam, and the other end was fastened with a pair of aluminum crimping parts. Meanwhile, the test was loaded by displacement control, with the moving velocity of the beam at 10 mm/min. By comparing the tensile stress-displacement curves of the crimped material during stretching under the action of different crimping parts with the same loading conditions and crimping amount, the advantages of the bionic crimping structure in terms of anti-slip performance would be highlighted (see Figure 10).

## 3. Results and Discussion

### 3.1. Effects of Bionic Crimping Structure on the Crimping Process

Figure 6 shows the resulting Mises stress in the crimping process for the bionic crimping structure and the traditional crimping structure. Compared with the traditional cusp-to-cusp crimping structure in Figure 6(b), the bionic cusp-to-fossa crimping structure in Figure 6(a) can effectively reduce the mechanical stress and stress concentration of the hose body to protect its structural strength and stability in the case of the same amount of crimping. This can be attributed to changes in geometric contact area as the sharpness of the crimping structure decreases [25]).

### 3.2. Effects of Bionic Crimping Structure on the Working Process

Figure 7 presents the resulting maximum principal strain in the working process for the bionic crimping structure in Figure 7(a) and the traditional crimping structure in Figure 7(b). It can be found that the strain/deformation at the cusp of the traditional structure is serious, causing the crimped materials to be at the risk of damage and slippage. When the crimped materials and the crimping parts have a relative movement tendency in the Y direction, the crimping parts will tend to be pushed in the direction perpendicular to this leading surface. Therefore, the traditional crimping parts with a negative rake structure in Figure 7(b) will be pushed apart in the X direction, whereas the bionic crimping parts with a positive rake angle in Figure 7(a) drive the body close to it [7].

Through the above analysis, it can be found that the cusp has an excellent penetrating capability, and the fossae functions to withhold and contain. The advantages of the cusp-fossae combination are obvious, which can not only reduce the force and energy required, facilitate the smooth progress for the crimping process, but also improve the anti-slipping stability of the crimping structure.

### 3.3. Experimental Analysis of the Anti-Slipping Performance of Bionic Crimping Structure

Figure 10 depicts the tensile stress-displacement curves of the crimped material, in which the end of the curve represents its slippage or fracture. As a polymer material, rubber exhibits a strict proportional relationship between stress and displacement when it is just stretched. If the elongation continues, the relationship between stress and displacement is still positively correlated, but no longer proportional and reaches a maximum at the yield point *d*. In the case of a small crimping amount of 0.2 mm (see Figure 10(a) and 10(b)), the stress of the experimental strip decreases when the strain exceeds the yield point until it slips out. However, the bionic structure significantly delays slippage of the material being crimped, and the corresponding tensile displacement extends from 75.317 mm to 170.637 mm, showing high resistance to slipping off compared with the traditional one. In the case of a large crimping amount of 1.0 mm (see Figure 10(c) and 10(d)), the microcrystalline structure in the test strip material was severely damaged, and its molecules did not have time to rearrange in the direction of force, showing brittleness. It was further found that the bionic structure has high crimping reliability and less damage to the material. The tensile strain increased by about 3.58%. The above results both suggest that the bionic crimping structure has a good comprehensive performance in terms of anti-slipping performance.

## 4. Conclusions

This work is dedicated to learning from the natural friction pair of ruminant molars for enhancing the anti-slipping performance of the crimping structure. Based on the similarity analysis of structure and function, the special infundibulum dentis structure was applied to the bionic design of the crimping structure. This study recommends the use of this novel designed bionic structure for the crimping process according to the following evidence given by computer simulation or physical experiment:

1. Taking the resulting Mises stress as an index of evaluation, the bionic crimping structure can reduce the mechanical stress and stress concentration of the hose body to protect its structural strength and stability in the simulation modeling of the crimping process.
2. Taking the resulting maximum principal strain as an index of evaluation, the material strain under the action of traditional structure is serious, causing the crimped materials to be at the risk of damage and slippage in the simulation modeling of the working process, whereas the bionic crimping structure cleverly improves this defect.
3. Compared with the traditional crimping structure, this bionic structure shows a higher level of resistance to slippage and reliability in a tensile test for the crimped material.

It contributes to an in-depth understanding of tooth morphology and provides new ideas for the design of biomimetic functional surfaces. Within the limits of our current research, the macrogeometry of ruminant molars was imitated. However, it still needs continuous exploration from effective bionics to high-performance bionics. Multicoupled bionics is a possible area for future investigation considering the excellent material properties of natural teeth.

## Figures and Tables

**Figure 1:** Schema of crimping structure.

**Figure 2:** Extraction of biological coupling elements of bovine molar.

**Figure 3:** Typical occlusal mode of natural teeth: (a) human teeth; (b) bovine molars; (c) wolf teeth.

**Figure 4:** CAD model reconstruction of bovine molar based on reverse engineering technology.

**Figure 5:** FEA simulation for crimping process: (a) meshing; (b) result data collection.

**Figure 6:** Resulting Mises stress in the crimping process for (a) bionic and (b) traditional crimping structures.

**Figure 7:** Resulting maximum principal strain in the working process for (a) bionic and (b) traditional crimping structures.

**Figure 8:** Tensile test platform for crimped material.

**Figure 9:** Detail drawing of simplified (a) bionic and (b) traditional crimping parts.

**Figure 10:** Tensile stress-displacement curves under the condition of (a) bionic structure, 0.2 mm crimping amount; (b) traditional structure, 0.2 mm crimping amount; (c) bionic structure, 1.0 mm crimping amount; (d) traditional structure, 1.0 mm crimping amount.

## Data Availability

All data generated or analyzed during this study are included in this published article.

## References

[1] Niu X., Hao G., Zhang C., Li L. (2021). Design and experimental verification of pressurized cylinders in hydraulic rubber hose pressure washers. *Actuators*.

[2] Wehlin C., Persson J., Ölvander J. (2020). Multi-objective optimization of hose assembly routing for vehicles. *Proceedings of The Design Society: Design Conference*.

[3] Smith J. D. (2018). Hose technology. *Rubber Products Manufacturing Technology*.

[4] Lee G. C., Kim H. E., Park J. W., Jin H. L., Lee Y. S., Kim J. H. (2011). An experimental study and finite element analysis for finding leakage path in high pressure hose assembly. *International Journal of Precision Engineering and Manufacturing*.

[5] Cho J. R., Jee Y. B., Kim W. J., Han S. R., Lee S. B. (2013). Homogenization of braided fabric composite for reliable large deformation analysis of reinforced rubber hose. *Composites Part B: Engineering*.

[6] Kwak S. B., Choi N. S. (2009). Micro-damage formation of a rubber hose assembly for automotive hydraulic brakes under a durability test. *Engineering Failure Analysis*.

[7] Evans A. R., Sanson G. D. (2003). The tooth of perfection: functional and spatial constraints on mammalian tooth shape. *Biological Journal of the Linnean Society*.

[8] Ungar P. S., Hartgrove C. L., Wimberly A. N., Teaford M. F. (2017). Dental topography and microwear texture in *Sapajus apella*. *Biosurface and Biotribology*.

[9] Tian K., Li X., Zhang B., Chen Q. (2017). Design and test research on cutting blade of corn harvester based on bionic principle. *Applied Bionics and Biomechanics*.

[10] Zhang Z., Wang X., Tong J., Stephen C. (2018). Innovative design and performance evaluation of bionic imprinting toothed wheel. *Applied Bionics and Biomechanics*.

[11] Wang J., Cheng C., Zeng X., Zheng J., Zhou Z. (2020). Bionic-tribology design of tooth surface of grinding head based on the bovine molar. *Tribology International*.

[12] Wang J., Cheng C., Chen Y., Yang D., Zheng J., Zhou Z. (2020). Transfer of functional structures from multiple bovine teeth to a multilevel grinding head via a biomimetic approach. *Tribology International*.

[13] Wolf M., Schulte U., Küpper K. (2016). Post-treatment changes in permanent retention. *Journal of Orofacial Orthopedics*.

[14] Xiao H., Lei L., Peng J. (2019). Research of the role of microstructure in the wear mechanism of canine and bovine enamel. *Journal of the Mechanical Behavior of Biomedical Materials*.

[15] Soana S., Gnudi G., Bertoni G. (1999). The teeth of the horse: evolution and anatomo-morphological and radiographic study of their development in the foetus. *Anatomia, Histologia, Embryologia*.

[16] Soana S., Bertoni G., Gnudi G., Botti P. (1997). Anatomo-radiographic study of prenatal development of bovine fetal teeth. *Anatomia, Histologia, Embryologia*.

[17] Vollmerhaus B., Roos H., Knospe C. (2002). The origin and function of the enamel cup, infundibulum dentis, on the incisors of the horse. *Anatomia, Histologia, Embryologia*.

[18] Weimer P. J., Hall M. B. (2020). The potential for biomimetic application of rumination to bioreactor design. *Biomass and Bioenergy*.

[19] Tsai M. T., Huang H. L., Yang S. G., Su K. C., Hsu J. T. (2021). Biomechanical analysis of occlusal modes on the periodontal ligament while orthodontic force applied. *Clinical Oral Investigations*.

[20] Lundqvist S., Haraldson T. (1992). Oral function in patients wearing fixed prosthesis on osseointegrated implants in the maxilla: 3-year follow-up study. *European Journal of Oral Sciences*.

[21] Zhang L., Liu Q., Zou D., Yu L. (2016). Occlusal force characteristics of masseteric muscles after intramuscular injection of botulinum toxin A(BTX - A)for treatment of temporomandibular disorder. *British Journal of Oral and Maxillofacial Surgery*.

[22] Che J., Zhang Y., Wang H., Liu Y., Suo C. (2021). A novel method for analyzing working performance of milling tools based on reverse engineering. *Journal of Petroleum Science and Engineering*.

[23] Li Z., Xiang H., Li Z., Han B., Huang J. (2013). The research of reverse engineering based on geomagic studio. *Applied Mechanics and Materials*.

[24] Fuentes F. J., Cordier J. J., Leonard P., Scherrer L., Popa T. (2019). Methodology for reverse engineering analysis of ITER as-built integrated systems. *Fusion Engineering and Design*.

[25] Rechberger M., Paschke H., Fischer A., Bertling J. (2013). New tribological strategies for cutting tools following nature. *Tribology International*.

